The article "Helicobacter bilis Contributes to the Occurrence of Inflammatory Bowel Disease by Inducing Host Immune Disorders" was published in 2022. Journal: Biomed Res Int.

# *Helicobacter bilis* Contributes to the Occurrence of Inflammatory Bowel Disease by Inducing Host Immune Disorders

**DOI:** 10.1155/2022/1837850

**Published:** 2022-08-09

**Authors:** Wei Peng, Xinhua Zhao, Xiaoan Li

**Affiliations:** Department of Gastroenterology, Mianyang Central Hospital, Sichuan, China 621000

## Abstract

Gut microbiota coevolve with humans to achieve a symbiotic relationship, which ultimately leads to physiological homeostasis. A variety of diseases can occur once this balance is disrupted. *Helicobacter bilis* (*H. bilis*) is an opportunistic pathogen in humans, triggering multiple diseases, including inflammatory bowel disease (IBD). IBD is a chronic immunologically mediated inflammation of the human gastrointestinal tract, and its occurrence is closely related to the gut microbiota. Several studies have demonstrated that *H. bilis* colonization is associated with IBD, and its mechanism is related to host immunity. However, few studies have investigated these mechanisms of action. Therefore, this article is aimed at reviewing these studies and summarizing the mechanisms of *H. bilis*-induced IBD from two perspectives: adaptive immunity and innate immunity. Furthermore, this study provides a preliminary discussion on treating *H. bilis*-related IBD. In addition, we also demonstrated that *H. bilis* played an important role in promoting the carcinogenesis of IBD and discussed its mechanism.

## 1. Introduction

The human gastrointestinal tract contains several groups of microorganisms, including bacteria, viruses, fungi, and archaea [1]. Among them, bacteria have been the most extensively studied, and a new genomic blueprint of the human gut microbiota has identified 1952 human gut bacteria [2]. Over the years, the rapid development of 16S rRNA-based technology has enhanced our understanding of complex ecosystems and gut microbiota diversity [3]. The human gut microbiota coevolved with humans to achieve a symbiotic relationship, leading to physiological homeostasis. During this interaction, several physiological conditions occur, such as the potential of hydrogen, redox potential, and transit time, change with different parts of the digestive tract, resulting in differences in the microbial community composition in the upper and lower digestive tract [4]. It has been suggested that the highest concentration and different types of bacteria comprising the gut microbiota of humans reside in the cecum and colon [5].

Several studies have proven that the gut microbiota is closely related to human diseases, such as inflammatory bowel disease (IBD), colon cancer, and metabolic syndrome [6–8]. Among them, IBD is the most extensively studied and has been shown that its pathogenesis is closely associated with gut microflora and immunity. Various mouse models of IBD include spontaneous colitis models, chemically induced colitis models, colitis in immunodeficient mice, genetically engineered models, or any combination of these models. Recently, a newly identified murine pathogen, *Helicobacter bilis* (*H. bilis*), has been related to gut infection causing chronic inflammation [9]. Therefore, *H. bilis* has been widely used to establish IBD mouse models in many studies, but the mechanism remains unclear [10]. This review will focus on the relationship between *H. bilis* and IBD and summarize its mechanism.

The article "Helicobacter bilis Contributes to the Occurrence of Inflammatory Bowel Disease by Inducing Host Immune Disorders" was published in 2022. Journal: Biomed Res Int.

### 1.1. Characteristics of *Helicobacter bilis*

*Helicobacter* spp. are gram-negative, microaerobic, helical-shaped bacteria that comprise more than 35 species [11, 12]. *Enterohepatic Helicobacter* spp. (including *Helicobacter canis*, *Helicobacter marmotae*, and *H. bilis*) colonize the hepatobiliary systems and intestinal tracts of various mammals [13]. *H. bilis* is an opportunistic, nonsporulating, and fusiform bacterium that has a fusiform body with 3–14 bipolar flagella and periplasmic fibers wrapped around the cell [14]. Furthermore, *Flavispira* spp. isolated from diarrheal humans and animals were reclassified as *H. bilis* [15]. 16S rRNA gene sequence analysis showed that *H. bilis* gene sequence was 98% similarity to *Helicobacter cinaedi* and 93.4% similarity to *Helicobacter pylori* (*H. pylori*) [16]. However, unlike *H. pylori*, *H. bilis* belongs to the *enterohepatic Helicobacter species*, which can grow in the bile and intestine but not in the stomach [14].

*H. bilis* possesses one of the broadest host spectra of the *Helicobacter* genus and can be found in humans and some animal species [17]. Isolation of *H. bilis* from the bile, liver, and intestines of aged inbred mice was first reported by Fox et al. in 1995, on the basis of 16S rRNA gene sequence analysis [16]. In humans, *H. bilis* was first detected via PCR in the gallbladder and bile of Chilean patients with chronic cholecystitis [18]. Importantly, through fluorescence in situ hybridization, our previous studies detected the presence of *H. bilis* in human IBD and colorectal cancer tissues [19].

As an opportunistic pathogen in humans, *H. bilis* colonization can trigger multiple gastrointestinal diseases such as IBD, hepatitis, cholangitis, colitis, and even malignancies [20, 21]. Among the *H. bilis*-induced malignancies, hepatobiliary carcinoma is most extensively studied, and the important role of *H. bilis* in MALT-associated gastrointestinal lymphomas was revealed by Woods and collaborators [14, 22]. In addition to digestive diseases, Chen et al. showed that *H. bilis* is also associated with neurological conditions such as Alzheimer's disease [23]. Of the diseases induced by *H. bilis*, IBD has received widespread attention. It has been confirmed that *H. bilis* is involved in the occurrence and development of IBD by inducing a host immune response.

The article "Helicobacter bilis Contributes to the Occurrence of Inflammatory Bowel Disease by Inducing Host Immune Disorders" was published in 2022. Journal: Biomed Res Int.

### 1.2. Inflammatory Bowel Disease

IBD includes Crohn's disease (CD) and ulcerative colitis (UC), which are chronic, immunologically mediated disorders of the human gastrointestinal tract [24]. CD is characterized by chronic inflammation of any part of the gastrointestinal tract, which can disrupt the mucosa or include healthy areas between affected sites [25]. A typical clinical scenario is an abdominal pain, chronic diarrhea, weight loss, and fatigue [26]. Patients with UC have mucosal inflammation starting in the rectum that can extend continuously to proximal segments of the colon; however, some patients with proctitis or left-sided colitis might have a cecal patch of inflammation [27, 28]. The clinical course of UC is unpredictable and is marked by alternating periods of exacerbation and remission. Worldwide, there is a trend towards an increasing incidence of both UC and CD. A recent systematic review showed that 75% on CD and 60% on UC confirmed a secular trend in the disease incidence [29]. IBD is one of the most intensely studied chronic inflammatory diseases, the etiology of which involves the environment, host genetics, host innate and adaptive immune components, and symbiotic microorganisms [30]. IBD is likely driven by aberrant immune responses directed against the resident microbiota [31, 32]. Susceptible IBD sites are also those with relatively high bacterial density, such as the distal ileum and cecum. Therefore, the occurrence and development of IBD are closely related to the gut microbiota.

Over the years, several studies demonstrated that the immune cells (including macrophages, T cells, and innate lymphoid cells) and pathogenic immune cell circuits are recognized as crucial drivers of IBD. For example, mucosal immune cells can respond to microbial products or antigens from the commensal microbiota by producing cytokines, and the overexpression of proinflammatory cytokines (such as IL-1, IL-2, IL-5, IL-6, IL-12, IL-18, and IFN-*γ*) can promote the development of IBD [33–35]. Conversely, anti-inflammatory cytokines (such as IFN-*β*, IL-10, and IL-11) or the neutralization of proinflammatory cytokines can prevent and treat chronic intestinal inflammation [36, 37].

### 1.3. *H. bilis* Promotes IBD through Inducing Aberrant Immune Responses in the Host

The intestinal immune system comprises of intestinal epithelial cells, intestinal intraepithelial lymphocytes, lamina propria lymphocytes, peyer patches, and gut-associated lymphoid tissue [38]. The immune system is involved in the maintenance of gut microbiota composition. On the other hand, the gut microbiota regulates and affects the innate and adaptive immune systems at multiple levels, and some studies have explored how some specific bacteria interact with the immune system [39]. The human immune system and gut microbiome interact to maintain homeostasis in the gut, and alterations in the gut microbiome composition lead to immune dysregulation, ultimately promoting chronic inflammation [40]. Ever since the late 1990s, the relationship between colitis and *H. bilis* has been recognized [41]. The histopathology of *H. bilis*-induced IBD includes crypt hyperplasia, inflammatory cell infiltrates, crypt abscesses, and obliteration of normal gut architecture. In this study, the relationship between *H. bilis* and IBD was established by searching in PubMed, MEDLINE, and Web of Science databases, and these results were shown in Table 1 [9, 41–53]. Some studies clarified how *H. bilis* promotes IBD occurrence and development; however, few studies have summarized these mechanisms. Therefore, in this review, we reviewed and classified the mechanisms mentioned in these studies.

1. Adaptive immune: the introduction of *H. bilis* may disrupt mucosal homeostasis and subsequently increase the host's susceptibility to IBD following an inflammatory event, and its mechanism may be related to significant increases in mucosal gene expression. *H. bilis* colonization could significantly increase the expression of numerous mucosal genes (e.g., Fut2, B3galt5, Ceacam12, Cyp4b1, and Ugt8a), which could lead to increased protein glycosylation and dysregulation of detoxification (Figure 1(a)). This increase in the expression levels can potentially predispose the host to the onset of colitis following a severe inflammatory insult, consistent with a “multiple-hit hypothesis” for the development of IBD [47]. In addition, Liu and collaborators found that genes associated with T cell activation (such as Cd28) and chemotaxis (such as Ccl8, Ccr5, and Itgb2) were significantly upregulated in mice receiving *H. bilis* (Figure 1(b)). These results suggest that *H. bilis* may alter mucosal homeostasis, promote immune cell activation and migration, and exacerbate the inflammatory response [46]

Some studies suggested that individual bacteria have a limited role in developing host disease, and they may play a pathogenic role by affecting the gut microbiome. This gregarious communication in the bacterial population is named quorum sensing (QS), which enables bacteria to feel their surrounding environment and to regulate their density and behavior via diffusible signal molecules called autoinducers (AIs) [54, 55]. AIs can affect intestinal epithelial cells and intestinal immune function, and intestinal epithelial cells and immune cells can also “listen” to the communication between bacterial communities and change the biological behavior of bacteria according to these signals [56, 57]. This interaction may be a potential target for gut bacteria to induce IBD through the immune pathway. Some studies have confirmed that *H. pylori* could produce AIs, such as N-acyl homoserine lactones and autoinducer-2, to influence spatial distributions of cells within a biofilm community [58]. So, could *H. bilis*, which is highly homologous to *H. pylori*, have a similar effect? Importantly, Atherly et al. showed that *H. bilis* infection could alter the distribution of resident intestinal mucosal bacteria in C3H/HeN mice, to induce host adaptive immune responses, leading to the occurrence and development of chronic intestinal inflammation [43]. In addition, this view has also been confirmed in other studies [48, 49]. We speculate that *H. bilis* affects bacterial quorum sensing by secreted autoinducer factors in the human intestine, resulting in structural changes of the gut microbiota, inducing host immune disorders, and thus activating its downstream inflammatory signaling pathway, eventually leading to the occurrence of IBD (Figure 1(c)). However, it is still unclear which autoinducer *H. bilis* secretes to participate in and regulate QS.

The article "Helicobacter bilis Contributes to the Occurrence of Inflammatory Bowel Disease by Inducing Host Immune Disorders" was published in 2022. Journal: Biomed Res Int.

However, Gomes-Neto et al. showed that *H. bilis* infection could induce severe intestinal inflammation in the presence of microbiota but did not alter the microbiota composition. The authors demonstrated that *H. bilis* colonization triggers CD4^+^ Th17 cell immunoreactivity against specific members of the resident microbiota but not toward itself. For instance, CD4^+^ T cells account for more than 60% of lymphocytes in the human gut [59]. Furthermore, evidence from a growing number of murine models of IBD supported a central role in dysregulated CD4^+^ T cell responses [60]. This result demonstrates that a synergistic effect between pathogenic factors and microbiota can exacerbate the inflammatory response in mice [42]. Finally, these reactions lead to the overexpression of proinflammatory cytokines (IL-6, IL-10, IL-12, IFN-*γ*, and TNF-*α*), which eventually leads to the development of IBD [51].

Interestingly, the potential virulence factors of *H. bilis* were first explored by Javed and collaborators [44]. Gamma-glutamyl transpeptidase is ubiquitous in all life forms and has implications for many physiological disorders [61]. Gamma-glutamyl transpeptidase produced by *Helicobacter pylori* (HPgGT) causes glutamine and glutathione consumption in host cells, ammonia production, and reactive oxygen species generation [62]. Similar to HPgGT, *H. bilis* releases a specific virulence factor (*H. bilis* Gamma-Glutamyl transpeptidase, HBgGT) to inhibit the activity of T cells. Subsequently, glutamine deprivation, total consumption of glutathione, and subsequent generation of free radicals by HBgGT can induce oxidative stress response cascades in colon epithelial cells (Figure 1(d)). Reactive oxygen species (ROS) activate the oxidative stress-associated signaling pathways, including NF-*κ*B, AP-1, and CREB, ultimately leading to the expression of the proinflammatory cytokine IL-8 [44]. During infection, IL-8 is secreted in response to infection and oxidative stress, recruiting inflammatory cells, and conversely, the IL-8 enrichment leads to an additional increase of oxidative stress mediators and inflammatory injury [63, 64]. Similarly, *H. bilis* has also increased ROS production in cholangiocytes, a risk factor for cholangiocarcinogenesis [65]. In addition to HBgGT, *H. bilis* can secrete other virulence factors, such as urease and cytolethal distending toxin [44]. However, the functions of these virulence factors during an *H. bilis* infection need to be explored.

(2) Innate immune: innate immune responses are formed under external antigen stimulation conditions, which can be quickly initiated and activated after infection to remove pathogens invading the human body. The innate immune system is considered a crucial cellular component of the chronic proinflammatory state of the gut during IBD. It comprises pattern recognition receptors (PRRs) and immune cells (including macrophages, dendritic cells, and neutrophils) that do not undergo somatic rearrangement [66]

Macrophages reside in the lamina propria and are principal innate immune effector cells that play an essential role in homeostasis [67]. Intestinal macrophage dysfunction is widely recognized as a central component IBD pathogenesis [68]. Muthupalani et al. suggested that macrophages are critical inflammatory cellular mediators that promote *H. bilis*-induced IBD in BALB/c mice, and the macrophage depletion promotes positive therapeutic effects in humans and experimental mice (Figure 1(e)) [45]. Furthermore, macrophages within the inflamed mucosa are derived mainly from circulating macrophages can secrete members of the IL-1 family (including IL-1*α*, IL-1*β*, IL-18, IL-33, IL-36, IL-37, and IL-38), and these cytokines are associated with proinflammatory signaling in the context of IBD via activation of the NF-*κ*B transcription factor pathway [69, 70]. Moreover, it has been described that IL-1*α* and IL-1*β* are critical drivers of inflammation and tissue damage in IBD [69]. For instance, Maggio-Price et al. demonstrated that *H. bilis* could increase the expression of the proinflammatory cytokines interleukin IL-1*β* and IL-1*α* secreted by macrophages and finally promote the development of IBD [50]. It is known that macrophages are modulators of the regulatory T cell population, and therefore, innate and adaptive immune cannot be separated during the pathogenesis of *H. bilis*-associated IBD.

The article "Helicobacter bilis Contributes to the Occurrence of Inflammatory Bowel Disease by Inducing Host Immune Disorders" was published in 2022. Journal: Biomed Res Int.

### 1.4. Treatment of *H. bilis*-Associated IBD

The current treatment of IBD mainly relieves symptoms, usually using anti-inflammatory drugs, 5-ASA, and general immunomodulatory drugs such as thiopurine and methotrexate. In addition, some new treatments, including anti-TNF, have also been used clinically [71]. However, the drug treatment effect is often limited and accompanied by side effects, and anti-TNF-*α* therapy may promote serious and opportunistic infections [72]. Therefore, treating intestinal pathogenic bacteria may bring a turning point for IBD treatment. Elucidating the pathogenic mechanism of *H. bilis* could improve the IBD treatment; although, no specific drug exists to eliminate *H. bilis.* Nowadays, some studies have explored novel treatments for *H. bilis*-related IBD. For example, Seamons and collaborators demonstrated that the ALDH1A enzyme could inhibit *H. bilis*-induced colitis by altering the *α*4*β*7 (a gut-homing integrin) expression on activated T cells [9]. The results of this study provide a new target for the IBD treatment, but its efficacy has only been confirmed in animal models, and further research is urgently needed.

Antibiotics are effective in subsets of patients with IBD, and most rodent colitis models suggest that inflammation does not occur in sterile environments [73, 74]. However, the gut of humans is an important reservoir for the development of antibiotic resistance genes because of the great abundance and diversity of gut microbiota [75]. A study performed by Gao and Fan conducted an antibiotic resistance analysis of *H. pylori* in 365 Chinese people and found that the resistance rates to clarithromycin, amoxicillin, fluoroquinolone, and tetracycline were 65.06%, 7.54%, 61.39%, and 20.37%, respectively [76]. Interestingly, Liu and Zhang found that goat milk intake might decrease the transfer potential of antibiotic resistance gene to pathogenic bacteria in the gut, thus reducing the abundance of pathogenic bacteria, such as *H. bilis* [75]. Therefore, changes in diet may have some therapeutic effect on the antibiotic resistance of pathogenic bacteria.

The article "Helicobacter bilis Contributes to the Occurrence of Inflammatory Bowel Disease by Inducing Host Immune Disorders" was published in 2022. Journal: Biomed Res Int.

### 1.5. The Relationship between *H. bilis* and Colitis-Associated Carcinogenesis and Its Possible Mechanism

Colitis-associated carcinogenesis (CAC) incidence is highly correlated with the severity, duration, and extent of IBD [77]. The microbiota has the potential to form an inflammatory microenvironment and vice versa, and inflammation may also affect the microbial composition. Intestinal carcinogenesis is driven by microbial enrichment, chronic inflammation, and intestinal immunomodulation [78, 79]. In 2010, Ericsson et al. demonstrated that *H. bilis* infection in Smad3(-/-) mice leads to the development of colitis-associated mucinous colonic adenocarcinoma, which is strongly correlated with the expression of Il-1b, Mip-1a, and Cd5 (RANTES) [80]. In 2013, Nguyen et al. pointed out that *H. bilis* is not only an important risk factor for the development of chronic intestinal inflammation in WASP-deficient mice but also for dysplasia and CRC [81]. However, the mechanisms by which *H. bilis* causes CRC remain to be elucidated.

Recently, our study demonstrated that *H. bilis* infection is associated with IBD-related CAC, possibly by promoting the T cell transformation into CD4^+^CD45RB^+^T cells and increasing the expression of the proinflammatory cytokine IFN-*γ* [19]. Furthermore, Wu et al. found, using high-throughput sequencing, that the presence of *H. bilis* in moderately and poorly differentiated CAC tissues was higher than in well-differentiated CAC tissues [82]. This result suggested that *H. bilis* colonization was not only associated with cancer occurrence but could also promote the deterioration of CRC tissues. Patients with *H. bilis-associated* CAC may have worse prognosis than those with sporadic colon cancer. However, the studies included in our review were correlation analyses, and further studies are required to identify the specific mechanisms by which *H. bilis* promotes CAC development.

## 2. Conclusions

The gut microbiota can affect the development of the host immune system, and at the same time, the host immune system can regulate the gut microbial composition in the gut. Multiple studies have shown that the colonization of *H. bilis* could lead to the occurrence and development of chronic intestinal inflammation, and its pathogenic mechanism was related to host immune disorder. In our study, we summarize the mechanism of *H. bilis*-induced IBD, taking into account two aspects, adaptive immunity and innate immunity, and demonstrate that impaired host immunity is a crucial factor in promoting the development of many health conditions. Although the treatment of *H. bilis*-related IBD is directed to relieve symptoms, some studies have proposed new treatment strategies for the pathogenic mechanism of *H. bilis* in animal models, and gene-targeted therapy for humans may be the focus of future research. Furthermore, we mentioned that *H. bilis* colonization could continuously promote the deterioration of tumor tissue and affecting the disease prognosis. Overall, although the pathogenic mechanism remains unclear, monitoring microbial colonization, such as *H. bilis*, provides a new target for the prevention and treatment of IBD and IBD-related CAC.

The article "Helicobacter bilis Contributes to the Occurrence of Inflammatory Bowel Disease by Inducing Host Immune Disorders" was published in 2022. Journal: Biomed Res Int.

## Figures and Tables

**Figure 1:** *H. bilis* promotes IBD through inducing aberrant immune responses in the host. (a) *H. bilis* colonization could increase the expression of numerous mucosal genes (e.g., Fut2, B3galt5, Ceacam12, Cyp4b1, and Ugt8a), which could lead to increased protein glycosylation and dysregulation of detoxification. (b) *H. bilis* colonization could increase the expression of genes associated with T cell activation and chemotaxis (e.g., Cd28, Ccl8, Ccr5, and Itgb2). (c) *H. bilis* affects bacterial quorum sensing by secreted autoinducer factors in the human intestine, resulting in structural changes of the gut microbiota. (d) *H. bilis* releases a specific virulence factor HBgGT to induce oxidative stress response cascades in colon epithelial cells. (e) *H. bilis* colonization could increase the expression of IL-1 family secreted by macrophages, and these cytokines are associated with proinflammatory signaling. *H. bilis*: *Helicobacter bilis*; ROS: reactive oxygen species; HBgGT: *H. bilis* gamma-glutamyl transpeptidase.

**Table 1:** *Helicobacter bilis*-induced inflammatory bowel disease.

Author	*H. bilis*	Research subjects	Mechanisms	Type of immunity	Year
Seamons et al. [9]	Not mentioned	Smad3^−/−^ mice	Not mentioned	Adaptive immunity	2020
Gomes-Neto et al. [42]	Not mentioned	C3H/HeN mice	Triggering CD4^+^ Th17 cell immunoreactivity against specific member of microbiota, but not toward itself	Adaptive immunity	2017
Atherly et al. [43]	ATCC strain 51630	C3H/HeN mice	Altering mucosal bacteria	Adaptive immunity	2016
Javed et al. [44]	ATCC strain 43879	Colon cancer cell lines HCT116 (CCL-247), DLD-1 (CCL-221), and LS174T (CCL-188)	HBgGT enhances inflammatory stress ROS in colon epithelial cells	Adaptive immunity	2013
Muthupalani et al. [45]	Not mentioned	BALB/c mice	Macrophages are critical inflammatory cellular mediators for promoting *H. bilis*-induced IBD	Innate immunity	2012
Liu et al. [46]	ATCC strain 51630	C3H/HeN mice	Altering mucosal homeostasis and initiating immune cell activation and migration	Adaptive immunity	2011
Liu et al. [47]	Not mentioned	C3H/HeN mice	Inducing mucosal gene expression changes	Adaptive immunity	2009
Jergens et al. [48]	ATCC strain 51630	C3H/HeN mice	Triggering persistent immune reactivity to antigens derived from the commensal bacteria	Adaptive immunity	2007
Jergens et al. [49]	ATCC strain 51630	C3H/HeN mice	Induction of differential immune reactivity to members of the flora	Adaptive immunity	2006
Maggio-Price et al. [50]	Not mentioned	Mdr1a^−/−^ mice	Increased expression of inflammation markers/mediators (MHC class II, Cox-2, CD4, F4/80) and monokine (IL-1*β*, IL-1*α*)	Innate immunity	2005
Maggio-Price et al. [51]	Provided by Dr. Lela Riley	Mdr1a^−/−^ and FVB mice	Cytokine dysregulation (IFN-*γ*, TNF-*α*, IL-10)	Adaptive immunity	2002
Burich et al. [52]	Provided by Dr. Lela Riley	C57BL mice	Not mentioned (correlation analysis)	Not mentioned	2001
Haines et al. [53]	Not mentioned	Male athymic nude rat	Not mentioned (correlation analysis)	Not mentioned	1998
Shomer et al. [41]	ATCC strain 51630	SCID mice	Not mentioned (correlation analysis)	Not mentioned	1997

HBgGT: *Helicobacter bilis* gamma-glutamyltranspeptidase; ROS: response via oxidative stress.
